# A Nomogram Model for Individualized Prediction of the Risk of Respiratory Tract Infection within Six Months after Diagnosis in Patients with Primary Immune Thrombocytopenia

**DOI:** 10.1155/2022/5002681

**Published:** 2022-07-28

**Authors:** Jinhua Wei, Weiwei Pan, Feng Luo, Fengnian Tang, Jiashi Wei, Siwen Fang, Honglian Huang

**Affiliations:** ^1^Department of Hematology, Department of Rheumatology and Immunology, The People's Hospital of Hechi, Hechi, 547000 Guangxi, China; ^2^Department of Gynecology, The People's Hospital of Hechi, Hechi, 547000 Guangxi, China

## Abstract

The risk factors of upper respiratory tract infection (URI) within 6 months after diagnosis in patients with idiopathic thrombocytopenic purpura (ITP) were analyzed, and the nomogram model was established and verified, with 242 and 50 ITP patients as the training and validation set, respectively. The patients were followed up for six months after the diagnosis of ITP. The clinical data of patients were collected, and the risk factors of URI in ITP patients within six months after diagnosis were analyzed using univariable, followed by multivariable logistic regression. Among the 242 ITP patients in the training set, 52 cases (21.49%) had URI, including 24 cases of viral infection, 11 cases of Mycoplasma pneumoniae infection, and 17 cases of bacterial infection. Logistic regression analysis showed that advanced age, use of glucocorticoid, smoking history, platelet count, serum CRP level, and lymphocyte subsets CD_4_^+^ and CD_8_^+^ were all risk factors for ITP patients to develop symptoms within six months after diagnosis (*P* < 0.05). Using the above five indicators, a nomogram prediction model was built for URI occurrence in patients with ITP within half a year after diagnosis, and the results showed an AUC, a sensitivity, and a specificity of 0.936 (95% CI: 0.878-0.983), 0.942, and 0.865, respectively. The nomogram model was internally verified by the bootstrap method for 500 self-sampling times, and the prediction of the calibration curve was in high consistency with the real results. External validation of the nomogram model resulted in an AUC, a sensitivity, and a specificity of 0.890 (95% CI: 0.757-0.975), 0.949, and 0.727, respectively. The nomogram model of URI in ITP patients within half a year after diagnosis based on logistic regression analysis has good discrimination and prediction accuracy. This provides important guidance value for individualized prediction of URI in ITP patients.

## 1. Introduction

Primary immunologic thrombocytopenic purpura (ITP) accounts for about 30% of all bleeding disorders [1], and its main clinical manifestations are decreased platelet count and severe bleeding. According to statistics, the global incidence of ITP was between 1.5 and 3.0‰ [2]. The incidence rate among adults in Europe was about 1.8‰ [3], and the incidence rate in China was 2.8‰ [4], which is higher than that in Europe. Glucocorticoids are the main drug treatment for ITP at present, but the risk of respiratory tract infection is high when taking the drugs [5]. It has been reported that the incidence of respiratory tract infection during treatment in ITP patients is as high as 5 times that of healthy people, and the mortality rate within 1 year of treatment is as high as 0.9%. The majority of deaths were from upper respiratory tract infection (URI) [6]. Therefore, while paying close attention to complications such as severe bleeding in ITP, we must also pay attention to the prevention and treatment of respiratory tract infections. At present, there is no analysis on the risk factors of URI in ITP patients within half a year after diagnosis; so, for ITP prevention and treatment, it is very important to identify relevant risk factors for URI within half a year after ITP diagnosis to screen out high-risk patients. How to realize the individualized prediction of the risk of ITP patients within six months after diagnosis is a difficulty that needs to be urgently solved, and there are few relevant reports at home and abroad.

A nomogram integrates relevant risk factors and visualizes risk values [7]. Based on this, this study analyzed the clinical data of ITP patients to explore the risk factors of URI within six months after diagnosis and built and validated a nomogram model for individualized prediction of URI risk in ITP patients within six months after diagnosis.

## 2. Materials and Methods

### 2.1. Study Population

A training set and a validation set, which included 242 ITP patients visited the Hechi People's Hospital between January 2019 and June 2020 and 50 ITP patients admitted between July 2020 and December 2020, respectively, were set up. Inclusion criteria for training and validation sets were as follows: (1) meet the clinical diagnostic criteria of “Chinese Expert Consensus on Diagnosis and Treatment of ITP in Adults 2016 Edition” [8], no less than two routine blood tests showed a decrease in platelet count, and bone marrow test showed an increase in the number of megacaryocyte and a mature disorder; (2) antibiotic treatment and splenectomy were performed after diagnosis; (3) those suffering from ITP for the first time; (4) age ≥ 18 years old; (5) the follow-up time is not less than six months; and (6) the patient voluntarily participated in this research with informed consent provided. Exclusion criteria were as follows: (1) patients with secondary thrombocytopenia; (2) patients treated with antiplatelet aggregation, anticoagulation, and other drugs; (3) patients with passive participation in this study; and (4) patients who were lost to follow-up and whose follow-up data were incomplete. The present study was a retrospective study.

### 2.2. Collect Patient Data

The Hospital Information System (HIS) was used to collect and summarize the clinical information of ITP patients on admission, including gender, age, drinking history (female drinking > 70 g pure alcohol/week, male > 140 g pure alcohol/week), smoking history (smoking more than 100 cigarettes or cumulative smoking of more than six months), pathogens, combined anemia, glucocorticoids, splenectomy therapy, rituximab, serum C-reactive protein (CRP) levels, natural killer (NK) cells, lymphocyte subpopulations CD_3_^+^, CD_4_^+^, CD_8_^+^, B lymphocyte, and platelet counts.

### 2.3. Grouping

All cases were followed up for half a year, and the follow-up was conducted in the form of outpatient review. Patients visited the hospital for reexamination every 1 month after discharge. According to the diagnostic criteria of acute upper respiratory tract infection [9], the patient had pharyngeal itching, dry throat, symptoms of upper respiratory catarrh or fever, headache, and other symptoms. Physical examination showed that the pharynx, nasal mucosa congestion, secretions, and edema were diagnosed as URI. The ITP patients in the modeling set who developed URI within half a year after diagnosis were assigned to the infected group, and those who did not were assigned to the uninfected group.

### 2.4. Statistics and Methods

SPSS 23.0 analyzed the original data. Continuous variables that obeyed the normal distribution were denoted by (mean ± standard deviation), and *t*-test conducted intergroup comparisons. The categorical variables was represented by *n* (%), and the chi-square test or rank-sum test conducted intergroup comparisons. Univariate and multivariate logistic regression were employed to identify prognostic factors of patients. URI risk in ITP patients within six months after diagnosis was analyzed using the logistic regression model, based on which a nomogram prediction model was built. The discriminative ability of the model was evaluated by calculating the area under the curve (AUC) and 95% confidence interval (CI), and internal validation with 500 iterations of bootstrap was used to evaluate the calibration effect through unreliability tests and calibration curves. *R* software (*v*4.1.2; https://www.r-project.org) was used. A *P* value <0.05 was interpreted as statistical significance.

## 3. Result and Discussion

### 3.1. Univariate Analysis of the Onset of Symptoms in ITP Patients within Half a Year after Diagnosis

Among the 242 ITP patients in the modeling set, 52 had URI, accounting for 21.49%, including 24 cases of viral infection, 11 cases of Mycoplasma pneumoniae infection, and 17 cases of bacterial infection. Statistically significant differences were present in age, use of glucocorticoid, smoking, platelet count, serum CRP level, and lymphocyte subsets CD_4_^+^ and CD_8_^+^ between infected and noninfected groups (*P* < 0.05), as shown in Table 1.

### 3.2. Multivariate Analysis of URI in Patients with ITP within Half a Year after Diagnosis

The dependent variable was the occurrence of URI (1 = yes, 0 = no) within six months after diagnosis of ITP patients, and the independent variables were the statistically significant features in Table 1. The categorical data was assigned a value (glucocorticoid application (1 = yes, 0 = no)), and the original value of the measurement data was entered. As indicated by the multivariate logistic regression analysis with results presented in Table 2, age, smoking history, glucocorticoid use, platelet count, serum CRP level, and lymphocyte subsets CD_4_^+^ and CD_8_^+^ were all risk factors for URI in patients with ITP within half a year after diagnosis (*P* < 0.05).

### 3.3. Establishment and Validation of the Risk Nomogram Model for URI in ITP Patients within Half a Year after Diagnosis

Seven independent risk factors obtained by logistic regression analysis were used for a nomogram model construction (Figure 1). Internal validation found that the predicted AUC, sensitivity, and specificity of the nomogram model for ITP patients with URI within six months after diagnosis were 0.936 (95% CI: 0.878-0.983), 0.942, and 0.865, respectively (Figure 2(a)). It suggests that the nomogram model has better discriminative ability. Hosmer-Lemeshow test for the deviation between the predicted value of the model and the actual value (chi − square = 14.249, *P* = 0.075) indicates that the prediction model has a good calibration ability. The mean absolute error (MAE) of the calibration curve from 500 samplings by the bootstrap method was 0.013, indicating that the occurrence risk predicted by model is in good agreement with the actual occurrence risk (Figure 2(b)).

The validation set (50 cases, of which 39 cases did not have upper symptoms and 11 cases of upper symptoms) was used to externally validate the model, and an AUC of 0.890 (95% CI: 0.757-0.975), a sensitivity of 0.949, and a specificity of 0.727 were determined (Figure 3(a)), demonstrating favorable prediction accuracy of the nomogram model. The calibration curve is close to the ideal curve, indicating that the predicted probability of the nomogram is basically consistent with the measured value (Figure 3(b)).

## 4. Discussion

With complex pathogenesis, ITP is generally believed to be linked to the reduction of platelet production and the excessive clearance of platelets by macrophages [10]. Studies have shown that [11], ITP patients with a history of respiratory tract infection in the first half of the month, the infection risk of ITP patients is much higher than that of the general population. Infection will increase the Fc and C3b receptors of macrophages, resulting in an increase in their affinity, and platelets are more easily destroyed [12]. ITP widely acknowledged to be associated with immune cell dysfunction and immune dysfunction [13]. Immune cell dysfunction and immune dysfunction are closely related to RTI [14]. However, the mechanism of the onset of symptoms in ITP patients within six months after diagnosis is unclear. Therefore, early and effective identification of ITP patients who are at risk of developing uppersensitivity is extremely important.

Among the 242 ITP patients, URI occurred in 52 cases, with an incidence rate of 21.49%, which was basically consistent with the results of domestic and foreign studies [15]. In this study, the age, using glucocorticoid, smoking, platelet count, serum CRP level, and lymphocyte subsets CD_4_^+^ and CD_8_^+^ were all influencing factors of ITP patients developing uppersickness within half a year after diagnosis. Elderly patients are often accompanied by other underlying diseases and may take a variety of drugs at the same time, resulting in a decline in body function and body resistance. Therefore, for elderly patients, follow-up should be strengthened, and preventive measures should be taken. For smokers, it is necessary to inform them of the dangers of smoking and instruct them to quit smoking. Because long-term smoking can easily lead to abnormal lung function in patients, the longer smoking time is, the easier it is to increase the risk of secondary respiratory tract infection in patients with ITP [16]. In the process of using glucocorticoid therapy, blood sugar will increase, which can cause the body's defense function to decline, and viruses and bacteria are more likely to invade the body at this time [17]. On the other hand, hormones can also affect the function of lymphocytes and monocytes, resulting in a decrease in the body's ability to resist infection, which leads to a greater susceptibility to upper feelings [18]. Kimura and Kishimoto [19] analyzed the medical records of 1805 ITP patients exposed to glucocorticoids and found that secondary respiratory infections were closely related to the recent use of glucocorticoids, and even low-dose applications had certain risks.

CRP level is an important indicator for judging URI. When the body is injured or infected, the level of CRP will rise rapidly, and it will fall back quickly after the patient's condition improves [20]. CRP levels in children with ITP are negatively correlated with platelet counts, and elevated CRP predicts lower platelet counts [21]. Kapur et al. [22] found a close association between CRP levels and antiplatelet antibodies in children's ITP. This study confirmed that elevated CRP was a risk factor for the development of upper-sensitivity. The dysfunction of T lymphocyte subsets is involved in the occurrence and development of URI, and its dysfunction and low immune function are closely related to URI [23]. T lymphocyte subsets are important indicators for judging the immune function of the body. Mature T lymphocytes can be divided into CD_4_^+^ and CD_8_^+^ subsets according to surface markers [24]. The synergistic effect of CD_4_^+^ and antigen stimulates B cells to secrete plasma cells, and the CD_4_^+^ T cells in some ITP patients are destroyed, resulting in decreased cellular immune function, which may increase the risk of URI [25]. In this study, the CD_4_^+^ level was statistically significant in the multivariate analysis, consistent with previous studies. CD_8_^+^ is a subset of cytotoxic cells or suppressor cells, an increase in the number indicates that the immune function is inhibited, and it is easy to cause a URI [26]. Platelets have a large number of receptor molecules on their surfaces, allowing them to rapidly sense invading pathogens and inflammation caused by infections [27]. Studies have shown [28] that respiratory tract infection is not only related to the immunomodulatory treatment of ITP patients but also to the platelet count of the disease itself. A compromised immune system can make patients more susceptible to infections before and after ITP develops. For bacterial infection, Gram-negative bacilli infection causes the release of endotoxin in the blood, which greatly enhances the phagocytosis of autoantibody-coated bacteria and accelerates the destruction of platelets [29]. For patients with low platelet levels, glucocorticoids, prednisone, dexamethasone, recombinant human thrombopoietin, and other drugs can be used for treatment. Doctors should adjust the treatment plan in a timely manner according to each patient's specific condition to ensure that the patient can get more benefits from the treatment.

Most of the previous research models are presented in the form of formulas, and the calculation process is complicated; not only there is the risk of calculation errors but also the workload of medical workers is increased. A good model should be effective, practical, and simple. The nomogram model can evaluate the prognosis intuitively, concisely, and accurately, which helps medical staff make better clinical decisions. Besides, the nomogram can uniquely reveal the correlation between relevant risk factors and outcome events [30]. In this study, a nomogram was built based on the abovementioned risk factors for URI in ITP patients within half a year after diagnosis, namely, age, corticoid application, smoking, serum CRP levels, and T lymphocyte subsets CD_4_^+^, CD_8_^+^, and internal verification was performed. The results showed that the model AUC = 0.936, sensitivity = 0.942, and specificity = 0.865 suggest that the nomogram model has better discriminative ability. After being verified by the validation set data, the predicted value of the model has a high consistency with the actual value, indicating that it has a good predictive ability. The limitation of this study is that this study is a single-center study, not a multicenter large-sample epidemiological survey. The data are from the same medical center, and there may be case selection bias. In the follow-up research work, this research group plans to cooperate with other centers to use its clinical data to further improve and improve the predictive value of the model.

## 5. Conclusion

Advanced age, use of glucocorticoid, smoking history, low platelet count, high CRP level, and low CD_4_^+^ and high CD_8_^+^ T cells were all risk factors for URI in patients with ITP within half a year after diagnosis. Based on logistic regression analysis, the nomogram model of the onset of symptoms in ITP patients within half a year after diagnosis has good discrimination and prediction accuracy. It can provide guidance for clinically accurate and personalized prediction of ITP patients.

## Figures and Tables

**Figure 1:** Nomogram model for predicting the risk of ITP patients to develop upper respiratory tract infection within half a year after diagnosis. CRP: C-reactive protein; CD_4_^+^: CD4-positive T-lymphocytes; CD_8_^+^: CD8-positive T-lymphocytes.

**Figure 2:** Internal verification of the nomogram model. (a) Risk of respiratory tract infection within six months after diagnosis in patients with primary immune thrombocytopenia by ROC curve. (b) Calibration curve of the nomogram model for training set. The *Y*- and *X*-axis represent the actual rate and the predicted risk of respiratory tract infection, respectively. The dotted line represents a perfect prediction made by an ideal model. The red line represents the actual model performance, and the closer it fits to the dotted line, the better the prediction.

**Figure 3:** External verification of the nomogram model. (a) ROC curve of model evaluation for validation set. (b) Calibration curve of the nomogram model for validation set. The *Y*- and *X*-axis represent the actual rate and the predicted risk of respiratory tract infection, respectively. The dotted line represents a perfect prediction made by an ideal model. The red line represents the actual model performance, and the closer it fits to the dotted line, the better the prediction.

**Table 1:** Single factor analysis that may affect the onset of symptoms in patients with ITP within half a year after diagnosis.

Clinical information	Noninfected group (*n* = 190)	Infected group (*n* = 52)	*χ* ^2^/*t*	*P*
Gender				
Male	112 (58.95)	26 (50.0)		
Female	78 (41.05)	26 (50.0)	1.334^b^	0.248
Age (years)	59.45 ± 8.45	64.85 ± 10.92	3.815^a^	<0.001
Drinking history				
Yes	56 (29.47)	20 (38.46)		
No	134 (70.53)	32 (61.54)	1.531^b^	0.216
Smoking history				
Yes	71 (37.37)	37 (71.15)		
No	119 (62.63)	15 (28.85)	18.858^b^	<0.001
Pathogen				
Virus	108 (56.84)	37 (71.15)		
Germ	82 (43.16)	15 (28.85)	3.482^b^	0.062
Combined anemia				
Yes	67 (35.26)	22 (42.31)		
No	123 (64.74)	30 (57.69)	0.871^b^	0.351
Use of glucocorticoid				
Yes	96 (50.53)	40 (76.92)		
No	94 (49.47)	12 (23.08)	11.557^b^	0.001
Splenectomy treatment				
Yes	56 (29.47)	12 (23.08)		
No	134 (70.53)	40 (76.92)	0.827^b^	0.363
CRP(mg/L)	3.19 ± 0.78	3.77 ± 0.85	4.659^a^	<0.001
CD_3_^+^ (%)	74.39 ± 9.78	72.88 ± 9.22	0.998^a^	0.319
CD_4_^+^ (%)	39.23 ± 6.59	34.74 ± 7.33	4.248^a^	<0.001
CD_8_^+^ (%)	27.88 ± 6.64	34.78 ± 6.95	6.573^a^	<0.001
Platelet count (×10^9^/L)	25.25 ± 5.24	21.20 ± 6.85	4.610^a^	<0.001

Note: CRP: C-reactive protein; CD_3_^+^: CD3-positive T-lymphocytes; CD_4_^+^: CD4-positive T-lymphocytes; CD_8_^+^: CD8-positive T-lymphocytes. ^b^ stands for *χ*^2^ test, and ^a^ stands for *t-*test.

**Table 2:** Logistic regression analysis of the onset of symptoms in ITP patients within half a year after diagnosis.

Variable	*β*	SE	Wald *χ*^2^	*P*	OR (95% CI)
Age	0.095	0.028	11.320	0.001	1.100 (1.041, 1.163)
Smoking history	2.078	0.526	15.616	<0.001	7.987 (2.850, 22.383)
Glucocorticoid	1.853	0.551	11.328	0.001	6.378 (2.168, 18.763)
Blood platelet count	-0.138	0.045	9.393	0.002	0.871 (0.797, 0.951)
CRP	0.892	0.308	8.399	0.004	2.441 (1.335, 4.462)
CD_4_^+^	-0.108	0.038	8.399	0.004	0.897 (0.833, 0.967)
CD_8_^+^	0.203	0.040	26.022	<0.001	1.225 (1.133, 1.324)

Note: CRP: C-reactive protein; CD_4_^+^: CD4-positive T-lymphocytes; CD_8_^+^: CD8-positive T-lymphocytes.

## Data Availability

The labeled dataset used to support the findings of this study are available from the corresponding author upon request.
